# Leukemia can be Effectively Early Predicted in Routine Physical Examination with the Assistance of Machine Learning Models

**DOI:** 10.1155/2022/8641194

**Published:** 2022-11-24

**Authors:** Cheng Yu, Yin-yin Peng, Lin Liu, Xin Wang, Qing Xiao

**Affiliations:** ^1^Department of Hematology, The First Affiliated Hospital of Chongqing Medical University, Chongqing 400016, China; ^2^College of Hohai, Chongqing Jiaotong University, Chongqing 400016, China

## Abstract

**Objectives:**

The diagnosis of leukemia relies very much on the results of bone marrow examinations, which is never generally performed in routine physical examination. In many rural areas even community hospitals and primary care clinics, the lack of hematological specialist and facility does not allow a definite diagnosis of leukemia. Thus, there will be a significant benefit if machine learning (ML) models could help early predict leukemia using preliminary blood test data in a routine physical examination in community hospitals to save time before a definite diagnosis.

**Methods:**

We collected the routine physical examination data of 1230 newly diagnosed leukemia patients and 1300 healthy people. We trained and tested 3 machine learning (ML) models including linear support vector machine (LSVM), random forest (RF), and XGboost models. We not only examined the accordance between model results and statistical analysis of the input data but also examined the consistency of model accuracy scores and relative importance order of model factors with regard to different input data sets and different model arguments to check the applicability of both the models and the input data.

**Results:**

Generally, the RF and XGboost models give more identical, consistent, and robust relative importance order of factors that is also accordant with the statistical analysis, while the LSVM gives much different and nonsense orders for different inputs. Results of the RF and XGboost models show that (1) generally, the models achieve accuracy scores above 0.9, indicating effective identification of leukemia, and (2) the top three factors that contribute most to the identification of leukemia include red blood cell (RBC), hematocrit (HCT), and white blood cell (WBC), while the other factors contribute relatively less.

**Conclusions:**

This study shows a feasible case example for early identification of leukemia using routine physical examination data with the assistance of ML models, which can be conveniently, cheaply, and widely applied in community hospitals or primary care clinics to save time before definite diagnosis; however, more studies are still needed to validate the applicability of more ML models to a larger variety of input data sets.

## 1. Introduction

Leukemias are a group of life-threatening malignant disorders of the blood and bone marrow [1]. Usually, leukemia could be either of the myeloid or lymphoid lineages and is classified as acute or chronic in nature. Chronic leukemias (CL) tend to have more mature cells and are rare in pediatric patients, and acute leukemias (AL), on the other hand, are typically less mature and commonly occur in patients of all ages and are potentially rapidly fatal if not readily treated [2].

The prognosis of AL is poor, and the death rate of AL is dramatically high. Its complications are usually life-threatening, and its treatment is generally complex [3]. Furthermore, the conditions are rapidly fatal if not treated although AL is usually initially highly responsive to chemotherapy [4]. However, physician-related delays in the diagnosis of leukemia have been shown to contribute to poor outcomes and higher mortality associated with the disease in low-income nations [5]. There is a high medical need to improve the outcome of leukemia patients.

Clinical diagnosis of leukemia is generally according to the cytomorphology, immunophenotyping, cytogenetics, and molecular genetics of the bone marrow and blood samples [6], which have specific requirements on corresponding test equipment and experienced experts. However, in many rural areas, community hospitals, or primary care clinics, qualified specialists, and test facilities are usually unavailable, and even in qualified hospitals, such tests are usually more expensive and more specific for suspected patients already showing symptoms. Thus, leukemia is often undiagnosed or delayed diagnosed, which consequently delays the treatment and worsens the outcome of patients.

In this case, early screening and treatment of leukemia patients in time can be very important. Certainly, a good solution for this task is to evaluate the health condition of individuals according to their regular physical examination data, which is complicated and difficult because it requires the experiences of physicians and careful subjective judgement of the complex relationships among various test parameters. In contrast, machine learning (ML) models are right designed to be expert at this task of determining complex relationships. They can handle even thousands of parameters, and they are able to detect and utilize their interactions [7–11], which is highly attractive to clinicians for disease diagnosis [12].

ML model is a practical and versatile choice for the early screening of diseases. It has achieved significant development and is successfully applied to a wide range of data-related problems [7]. For example, in some studies, an unsupervised was used to predict the defluorination of per- and polyfluoroalkyl substances [13], a variety of ML models were used to make predictions, extract feature importance, detect anomalies, and discover new materials or chemicals [14], and also in medicine, ML models are used to help understanding and overcoming of diseases [8–11]. Traditionally, diagnostic test data of patients are artificially interpreted by experienced clinicians according to their expertise, whereas ML models try to automatically learn the expertise of these experiences, for the initial diagnosis [15], prognosis estimation of treatment complications [16], and even for the relapse monitoring [17]. ML models have been shown on par with experts in a variety of tasks in hematologic malignancies [10], including the diagnostic and therapeutic evaluation of leukemia [18, 19], such as the image recognition of blood smears for diagnosis and classification of leukemia [20, 21], or the automatic detection of acute leukemia using blood images [22]. Currently, more ML applications for the diagnosis of leukemia are using images of bone marrow or peripheral blood cells [20–27]. The practical attempts on its application of early screening of leukemia using preliminary health records, like routine laboratory blood test results, are much fewer [18]. Leukemia screening using primary routine physical examination is of significant benefit because no other data are required than those acquired in a regular physical examination, so large-scale general screening of leukemia in people is thus possible.

In this study, we aimed to try utilizing ML models for the early diagnosis of leukemia using only the individual routine medical examination results. The advantage of doing this is thus ML models can be conveniently, cheaply, and widely applied in community hospitals or primary care clinics and can save time as much as possible before disease progression. We hope this work could provide a feasible case example of using ML models to early screen leukemia patients.

## 2. Materials and Methods

### 2.1. Data Collection

The ML models require both training and test data. In this study, we employed the routine laboratory test results of blood samples of both leukemia patients and healthy people to train and test the ML models. The routine laboratory records of blood samples were collected from the database of the first affiliated hospital of Chongqing Medical University, including those of the leukemia patients from the department of hematology admitted during 2014.4∼2020.6 and those of healthy people from the physical examination center during 2020.1∼2020.6. The data collection was performed under the approval of their Medical Ethics Committee (Number: 2021-152), according to the principles of the Declaration of Helsinki. Besides the blood test records of the leukemia patients, we collected their personal information and medical histories as well. As it is very common for leukemia patients to receive treatment repeatedly, we kept only the blood records at their first admission to our hospital but waived those afterwards. Moreover, we double-checked their medical histories to exclude those patients who were already diagnosed and treated before in other hospitals.

After those efforts, we screened out totally 1230 identified leukemia patients, and accordingly 1230 blood records, with totally 284 parameters tested at least once. The largest number of tested parameters appearing in a single record is 134, while most records contain around 50 tested parameters. These blood test records of leukemia patients were scheduled to be the target group in the ML models.

For the control group of ML models, we randomly selected 1300 blood records of healthy people from the physical examination center of our hospital. Their medical histories were also checked to ensure they were not leukemia patients, but even so, strictly speaking, we did not exclude those who had been with leukemia but were not diagnosed yet. Hopefully, such probability is very limited. The blood test records of healthy people contain fewer tested parameters than those of the leukemia patients. Therefore, we had to keep only the intersection of their tested parameters (30 parameters in common) into the following steps (column 2 of Table 1).

### 2.2. Handling the Missing Values

In the healthy group, all records contain all the 30 tested parameters, but this is not true in the patient group, where about 2/3 of the patients' records are incomplete (Figure 1).

As some ML models can only handle data in form of the complete matrix, thus for dealing with those blanks in the record-parameter matrix, we could either fill blanks with estimations or directly drop those incomplete records. In order to evaluate the practicability of ML models, we designed 5 scenarios *A–E* according to the amount of records we kept in modeling (Figure 1). Scenario *E* keeping the most records also contains the most uncertainties, while scenario *A* with the fewest records is, however, the most accurate. The blanks in complete records were estimated as the mean of values in all other records containing the corresponding parameter.

During modeling, the total input data set of each scenario would contain the data of the leukemia patients of that scenario, and also, the data of the same number of healthy people randomly selected from the total 1300 healthy people.

### 2.3. Statistical Analysis

According to the 1230 records of patients and 1300 records of healthy people, means and standard variations (SD) of the 30 tested parameters were calculated (Table 1), using mean(), *sd*(), and *t.*test() functions in R language version 4.0.3 for Mac. Parameters were compared, and the *p* values show their different significance.

### 2.4. Machine Learning Model Selection and Construction

ML models have significant benefits for the preliminary screening of diseases. However, generally, it is hard to say which model is absolutely the best, because model applicability depends on specific data set. Usually, in practice, various models will be tested, and their results will be examined to determine which model performs the best.

In this study, we chose 3 ML models to be tested and examined: linear support vector machine (LSVM), random forest (RF), and XGboost models. The main reason for choosing them is because they are relatively much more popular and have shown good performance in various applications, and also because they are able to give relative importance to model input factors as well.

We utilized the very popular scikit-learn (sklearn) package (version 0.24.2 in Python 3.9 for Mac) [28] for LSVM and RF models and referred to the official XGboost code (version 1.5 for Mac in Python) for the XGboost model [29], which was called in sklearn via an API function *XGBClassifier*() of package *xgboost* in Python.

### 2.5. Model Results Examination

As the applicability of each ML model depends on specific data set, their model results have to be examined to check their applicability. Practically, firstly, a reliable model should show consistency and robustness with regard to its input data, and secondly, its result should be accordant with the results of other analysis method like statistical analysis as well.

Since the model input data of this study mainly depend on the scenario selection (see Section 2.2) and the split ratio which splits the total data into train and test subsets inside ML models, we prepared various input data sets with regard to different scenarios and different split ratios (*R*_train/total_ = 0.25,0.5,0.75), and accordingly, their results, including the scores of score() function of sklearn which returns the accuracy of the model on input data [28], the area under the curve score (*S*_auc_), as well as the relative importance order of model factors (order of contribution weight of specific factor to the model), would all be examined to check their consistency with regard to various input data sets.

## 3. Results

### 3.1. Statistic Results

As shown in Table 1, target records have significantly lower mean hematocrit (HCT), hemoglobin (HGB), red blood cell (RBC), etc., but significantly higher mean white blood cell (WBC), the percentage of neutrophils (NEUT%), etc., (*p* < 0.001 for all unadjusted comparisons). According to the *p* values, most of the parameters show a significant difference between the two groups, and generally, the HCT, HGB, and RBC show the most significant differences among those parameters.

Although the *p* values of many parameters show significant statistical differences between patients and healthy people, for a certain individual, it is hard to diagnose a person with leukemia or not only according to a single or even two parameters, because many values of the parameters of the patients still lie in its reference range. Thus, for diagnosis, more parameters need to be taken into consideration, which requires the determination of more complicated interrelationships behind. That's exactly what ML models are adept in.

### 3.2. Model Consistency Examination

During modeling, the argument *lambda* of the XGboost model and the argument *C* of the LSVM model were adjusted to suppress overfitting, and the model performance indicators including the accuracy scores on both train and test subsets (*S*_train_, *S*_test_) and the *S*_auc_ were collected in Tables 2–4. The accuracy scores and *S*_auc_ suggest all models have achieved good results because generally, the accuracy scores are mostly above 0.9 even when the *R*_train/total_ is 0.25. Among scenarios, the accuracy scores are higher under scenario *A*, indicating the filling of missing values induces more uncertainties than discarding incomplete records.

For checking model result consistency, although the accuracy scores in Tables 2–4 look very consistent, we still need to look into the relative importance order of model factors of the models, a typical result of which was shown in Figure 2. Results show that the importance order of the RF and XGboost models is generally accordant and insensitive to the input data and the overfitting suppression factor *lambda*. However, the importance order of the LSVM model is much different and is much more sensitive to the input data and the overfitting suppression factor *C*.

Moreover, the top 3 important model factors of the RF and XGboost models are the count of RBC, HCT, WBC, while the top 3 of the LSVM model are absolute lymphocyte count (LYM^#^), percentage of monocytes (MONO%), and NEUT% (Figure 2). Obviously, the results of RF and XGboost models are more accordant with that of the statistical analysis (see Section 3.1).

### 3.3. Top Model Factors Contributing to the Classification of Leukemia

By accepting the results of RF and XGboost models, the top 3 model factors that contribute most to the identification of leukemia patients are found to be the count of RBC, HCT, and WBC. The other factors contribute relatively less to the models.

## 4. Discussions

The clinical diagnosis of leukemia is primarily based on laboratory blood and bone marrow tests, but even the most skilled hematologist may overlook patterns, deviations, and relations between the increasing numbers of blood and bone marrow parameters that modern laboratories measure. In contrast, ML algorithms can easily handle hundreds of attributes (parameters), and they are capable of detecting and utilizing the interactions among these numerous attributes, which makes this field of medicine particularly interesting for ML applications [12].

Nowadays, ML has already been proven to be a versatile, precise, and robust tool in the diagnostic evaluation of leukemia [18]. Rehman et al. [30] proposed a robust segmentation and deep learning techniques with the convolutional neural network to train the model on the bone marrow images to diagnose acute lymphoblastic leukemia with 97.98% accuracy. Kumar et al. [31, 32] presented an automated detection system for the diagnosis of acute leukemia. The method implemented uses basic enhancement, morphology, filtering, and segmenting techniques to extract the region of interest using a k-means clustering algorithm. The proposed algorithm achieved an accuracy of 92.8% and is tested with the nearest neighbor and Naïve Bayes classifier on the dataset of 60 samples. Dese et al. [20] used 250 clinical images of blood smears acquired from Jimma University Specialized Hospital and a standard online database to develop an image query system for diagnosing leukemia, and its type with the accuracy is 97.69%. Loey et al. [32, 33] proposed an AML classification system that enhanced image contrast and extracted five features. An SVM classifier performed the classification. Experiments on a data set of 50 images produced 93.5% classification accuracy.

As most of the ML application on leukemia diagnosis was dealing with the microscopic images and flow cytometry of bone marrow or peripheral blood cell, there is a lack of early prediction ML model for leukemia based on routine laboratory results. In this study, the required data for the ML models we used are able to be commonly acquired from the very primary routine physical examination in the rural area, community hospitals, or primary care clinics, which could help the early recognition of leukemia.

As the applicability of a certain ML model depends upon specific input data set, in this study, three models including the LSVM, RF, and XGboost models were selected, and their results were examined to check their applicability. The reason for choosing them is because they are relatively more popular, and more importantly, the sklearn toolkit we employed could look into the relative importance (or say contribution weight) of each model factor to the model, from which we could both examine the most model details and find the top factors that play key roles in the recognition of leukemia. Another consideration is that these three models require relatively much less input argument during the model construction because more arguments usually lead to higher model sensitivity to these input arguments. Specifically, for the LSVM model, only the overfitting suppression factor *C* (adjusted during modeling) is specified, and for the RF model, only the number of trees (we set *n_*estimators = 200) is set, and for the XGboost model, only the learning rate (we set learning_rate = 0.05) and the overfitting suppression factor *lambda* (adjusted during modeling) are required. Results show that the RF and XGboost model achieved very good consistency and robustness because their results turned out consistent and are accordant with the statistical analysis. As for the bad result of the LSVM model, we would like to regard the reason relevant to the limitation of its linear kernel to its applicability in this case of our study, but we did not check further into it.

In order to deal with the missing values of the incomplete records, we checked the difference between rather discarding the incomplete records and filling the missing values with an estimated average of existing values. Results show that the filling of missing values using estimations tends to introduce more uncertainties than directly discarding these incomplete values. This is interesting because, in other literature, many authors follow the filling method without any discussion or examination. We believe that the difference between filling and discarding should be case-dependent, and we should pay more attention to dealing with missing values.

The results of the RF and XGboost models also show that in this study, the accuracy scores are generally at least above 0.9 on both the train and test subsets even when the train data are a quarter of the total input. This might be partly relevant to the capability of the RF and XGboost models and partly be relevant to the accuracy and specificity of the input data as well, because the data we collected are from either very healthy people or from relatively severe patients. Therefore, about the methodology of this study, more further work is actually still needed to check the applicability of more ML models including SVM and other ML models to a larger variety of data sets.

The top 3 model factors that contribute most to the recognition of leukemia are the count of RBC, HCT, and WBC. The other factors contribute relatively less to the models.

The result about the WBC's count sounds reasonable that, as leukemia is a blood cancer that usually begins in the bone marrow and leads to the overproduction of abnormal WBC [34], the inspection of blood cells under a microscope allows for the evaluation and diagnosis of diseases like leukemia [35]. WBC, as one of the main cell types in peripheral blood, plays important role in the immune system and is a main defense of the body against infections and diseases [27]. Normally, WBC grows in accordance with the body's need, but in the case of leukemia, they have generated abnormally and inefficiently [27]. As early as the early 1800s, the excess WBC count had been observed with the presence of leukemia [36]. However, leukocytosis is neither sufficient nor necessary for the diagnosis of leukemia, because on the one hand, leukocytosis is very common in infections, and on the other hand, leukemia patients sometimes have normal or even lower total WBC counts [3]; thus, leukemia cannot be judged only by the counts of WBC.

It also makes sense about the count of RBC and HCT. The RBC, transporting oxygen and carbon dioxide [27, 37], may probably modulate the activity of immune cells within their microenvironment as well [38, 39] and is known highly correlated to the HCT [40]. Because leukemia is the overexcessive proliferation of abnormal cells in the bone marrow and then inhibits the normal hematopoietic cells, it can be inferred the RBC and HCT might be normal in the early stage of leukemia and then decrease with the progression of RBC breakdown. Therefore, the count of WBC, RBC, and HCT might be potential indication markers associated with the development of leukemia and is probably also associated with other parameters like thrombocytocrit (PCT). But it does not mean only these three factors indicate leukemia, and the other factors are negligible, and actually, the other factors also contribute and should be taken into consideration as well in the ML modeling.

Good results have the ML models get. Although it should also be emphasized that the results of ML models can only be an auxiliary reference but have no opportunities to replace the definite diagnosis by physicians, the real advantage of ML models is that the ML models can be conveniently and widely applied in the routine physical examination in community hospitals or primary care clinics without much extra expense and can save much of the time before disease progression, because if the routine physical examination result of somebody was classified by ML models as potential leukemia in time, he would be suggested to visit specialized hematology physicians as soon as possible for a specialized examination.

## 5. Conclusions and Limitations

In this study, we conducted a retrospective case study of utilizing the ML models to help early diagnosis of leukemia using only preliminary blood test data from the routine physical examination at community hospitals or primary care clinics. We collected data of preliminary blood test of both newly diagnosed leukemia patients and healthy people to construct the train and test data sets for ML models. We selected three models including LSVM, RF, and XGboost models according to their popularity, application convenience, and their ability to tell the relative importance or contribution weight of each factor to the model. We examined the sensitivity of model results, including the accuracy score, the area under the curve score, and the importance order, to the model input data and model argument including the scenario selection, split ratio, and the overfitting suppression coefficient.

Results show that although the LSVM expressed very bad applicability to the input data of this study, the RF and XGboost turned out of good consistency and robustness with regard to the input data and model argument, and their results are also accordant to the result of statistical analysis of the collected data. Generally, the RF and XGboost models could achieve an overall accuracy score above 0.9 for all the input data we used in this study. The top three model factors that contribute most to the recognition of leukemia are the count of WBC, HCT, and RBC, and the other factors contribute relatively less.

This study is a feasible case example to show that leukemia can be early predicted using preliminary blood test data from routine physical examination with the assistance of ML models. The advantage of doing this is thus ML models can be conveniently, cheaply, and widely applied in community hospitals or primary care clinics and can save time as much as possible before disease progression. Nevertheless, the results of ML models cannot replace but still require the definite diagnosis of hematology physicians.

Technically, there are still a few limitations of this study that affect the confidence of our models: (1) the details about the applicability of ML models to our input data set are still not fully understood; (2) all records were retrospectively collected from the First Affiliated Hospital of Chongqing Medical University, which may cause selection bias; (3) there are potential uncertainties, including uncertainties of laboratory measurements or the possibility of undetected leukemia patient in the healthy group; (4) only 30 parameters are kept in the modeling procedure, while some other parameters dropped might also be a potential indicator of leukemia. Therefore, the result of this study shows a good case for early predicting leukemia using preliminary blood test data from routine physical examination with the assistance of ML models; however, further investigation and prospective studies are still needed in the future to validate the applicability of more ML models to a larger variety of input data sets.

## Figures and Tables

**Figure 1:** Distribution of the number of tested parameters in the records of patients. Five scenarios were designed containing different amount of records according to the amount of missing values.

**Figure 2:** Model factor importances of the XGboost and random forest models (a) and linear SVM model (b) when *R*_train/test_ = 0.75/0.25 on scenario *A*.

**Table 1:** Statistical analysis of tested parameters in patients and healthy people.

	Parameter	Mean ± SD in healthy people	Mean ± SD in patients	*P* of *t*-test	Unit	Reference value
1	WBC	6.36 ± 1.64	64.43 ± 104.56	1.75*e* − 65	10^9^/L	3.5∼9.5
2	RBC	4.85 ± 0.51	2.83 ± 1.03	∼0	10^12^/L	4.3∼5.8
3	HGB	148.40 ± 16.01	87.51 ± 29.43	∼0	g/L	130.0∼175.0
4	HCT	44.19 ± 4.18	26.70 ± 8.86	∼0	%	40.0∼50.0
5	MCV	91.34 ± 5.73	95.66 ± 9.22	2.98*e* − 43	fl	82.0∼100.0
6	MCH	30.66 ± 2.31	31.33 ± 3.31	2.59*e* − 9	pg	27.0∼34.0
7	MCHC	335.50 ± 10.80	327.56 ± 16.83	1.51*e* − 43	g/L	316.0∼354.0
8	PLT	215.94 ± 57.70	151.95 ± 299.73	4.98*e* − 12	10^9^/L	85.0∼303.0
9	PDW	14.80 ± 3.03	13.56 ± 3.47	1.09*e* − 19	fl	10.0∼18.0
10	MPV	11.50 ± 1.20	10.88 ± 1.31	3.40*e* − 31	fl	7.6∼13.2
11	PCT	0.25 ± 0.05	0.20 ± 0.36	8.64*e* − 4	%	0.1∼0.5
12	NEUT%	57.10 ± 8.21	30.65 ± 25.04	5.09*e* − 157	%	40.0∼75.0
13	LYM%	33.24 ± 7.59	23.24 ± 23.90	1.42*e* − 34	%	20.0∼50.0
14	MONO%	6.61 ± 1.74	5.85 ± 9.92	1.98*e* − 2	%	3.0∼10.0
15	EO%	2.52 ± 2.15	1.02 ± 2.31	7.65*e* − 61	%	0.4∼8.0
16	BASO%	0.53 ± 0.30	1.10 ± 2.81	8.36*e* − 10	%	0∼1.0
17	NEUT#	3.67 ± 1.28	20.61 ± 43.18	2.12*e* − 30	10^9^/L	1.8∼6.3
18	LYM#	2.07 ± 0.59	7.48 ± 25.86	3.78*e* − 10	10^9^/L	1.1∼3.2
19	MONO#	0.42 ± 0.15	1.71 ± 4.42	1.06*e* − 17	10^9^/L	0.1∼0.6
20	EO#	0.16 ± 0.15	0.84 ± 3.09	4.74*e* − 11	10^9^/L	0.02∼0.52
21	BASO#	0.03 ± 0.02	1.25 ± 4.10	1.60*e* − 18	10^9^/L	0∼0.06
22	RDW-CV	12.90 ± 1.02	16.53 ± 2.89	4.41*e* − 224	%	12.0∼16.0
23	P-LCR	37.00 ± 9.47	31.14 ± 10.37	1.40*e* − 44	%	10.0∼60.0
24	TP	75.47 ± 4.03	68.62 ± 8.77	4.75*e* − 105	g/L	63∼82
25	ALB	48.39 ± 2.95	38.97 ± 6.11	2.80*e* − 279	g/L	35.0∼50.0
26	TBIL	13.44 ± 5.19	12.96 ± 10.03	1.44*e* − 01	*μ*mol/L	3.0∼22.0
27	ALT	24.55 ± 17.42	40.20 ± 64.34	3.14*e* − 14	U/L	21.0∼72.0
28	AST	23.35 ± 9.45	40.53 ± 63.63	2.11*e* − 17	U/L	17.0∼59.0
29	UA	340.79 ± 88.96	367.93 ± 162.09	1.87*e* − 7	*μ*mol/L	208.0∼506.0
30	Cre	67.10 ± 15.83	77.96 ± 54.91	9.33*e* − 9	*μ*mol/L	58.0∼110.0

**Table 2:** Accuracy scores of model performances on different scenarios, train-set/test-set ratios, and regularizations. (*S*_train_ and *S*_test_ are accuracy scores of models on train data subset and test data subset respectively according to the *score()* function of sklearn; *S*_auc_ is the area under the curve score of model according to the *roc_auc_score()* function of sklearn; *R*_train/total_ is the ratio of train data to the total data) for random forest model.

*R*_train/total_	Scenario	*A*	*B*	*C*	*D*	*E*
0.75	*S*_train_	1	1	1	1	1
	*S*_test_	0.9951	0.9878	0.987	0.9834	0.9844
	*S*_auc_	0.9855	0.9747	0.9779	0.9797	0.9808

0.5	*S*_train_	1	1	1	1	1
	*S*_test_	0.9949	0.9871	0.9855	0.9816	0.9855
	*S*_auc_	0.9859	0.9744	0.9745	0.9767	0.9808

0.25	*S*_train_	1	1	1	1	1
	*S*_test_	0.9956	0.9851	0.9899	0.9869	0.9822
	*S*_auc_	0.9886	0.9692	0.9836	0.9803	0.9755

**Table 3:** Accuracy scores of model performances on different scenarios, train-set/test-set ratios, and regularizations. (*S*_train_ and *S*_test_ are accuracy scores of models on train data subset and test data subset respectively according to the *score()* function of sklearn; *S*_auc_ is the area under the curve score of model according to the *roc_auc_score()* function of sklearn; *R*_train/total_ is the ratio of train data to the total data) for random forest model for XGboost model (lambda is the overfitting suppression factor).

*lambda*	*R*_train/total_	0.75					0.5					0.25				
	Scenario	*A*	*B*	*C*	*D*	*E*	*A*	*B*	*C*	*D*	*E*	*A*	*B*	*C*	*D*	*E*
0.1	*S*_train_	0.9985	1	1	1	1	1	1	1	1	1	1	1	0.9995	1	1
	*S*_test_	0.9917	0.9878	0.9844	0.9818	0.9873	0.992	0.9898	0.9855	0.9863	0.9899	0.9956	0.9946	0.9899	0.9881	0.9866
	*S*_auc_	0.9806	0.9814	0.9778	0.9801	0.9851	0.9753	0.9823	0.9737	0.9829	0.9869	0.9886	0.987	0.9836	0.9834	0.9812

1	*S*_train_	0.9985	0.9986	0.9987	1	1	0.9992	0.9993	0.9987	0.9988	0.9988	0.9995	0.9991	0.9983	1	0.9992
	*S*_test_	0.9922	0.9869	0.9832	0.9822	0.9873	0.992	0.9892	0.9823	0.9851	0.9872	0.9956	0.9892	0.9886	0.9845	0.9811
	*S*_auc_	0.9823	0.9792	0.9764	0.98	0.9851	0.9753	0.9806	0.9708	0.982	0.9832	0.9886	0.9789	0.9811	0.9763	0.9738

10	*S*_train_	0.9985	0.9946	0.9949	0.994	0.9955	0.9985	0.9959	0.9949	0.9952	0.9961	0.999	0.995	0.9953	0.996	0.9974
	*S*_test_	0.9922	0.9856	0.9828	0.9814	0.9836	0.992	0.9865	0.9823	0.9816	0.9861	0.9942	0.9865	0.9886	0.9834	0.9766
	*S*_auc_	0.9794	0.9724	0.9735	0.9772	0.9802	0.9775	0.9714	0.97	0.9755	0.9824	0.9833	0.9724	0.9827	0.9743	0.9689

**Table 4:** Accuracy scores of model performances on different scenarios, train-set/test-set ratios, and regularizations. (*S*_train_ and *S*_test_ are accuracy scores of models on train data subset and test data subset respectively according to the *score()* function of sklearn; *S*_auc_ is the area under the curve score of model according to the *roc_auc_score()* function of sklearn; *R*_train/total_ is the ratio of train data to the total data) for random forest modelfor linear SVM model (*C* is the overfitting suppression factor).

*C*	*R*_train/total_	0.75					0.5					0.25				
	Scenario	*A*	*B*	*C*	*D*	*E*	*A*	*B*	*C*	*D*	*E*	*A*	*B*	*C*	*D*	*E*
0.01	*S*_train_	0.8449	0.7935	0.771	0.8234	0.8687	0.871	0.8805	0.915	0.917	0.9293	0.9231	0.9136	0.9262	0.9225	0.9365
	*S*_test_	0.8614	0.7999	0.7668	0.8297	0.8854	0.8841	0.8772	0.8943	0.9087	0.9182	0.9334	0.9137	0.9119	0.9135	0.9288
	*S*_auc_	0.5	0.5	0.5479	0.7141	0.8315	0.5767	0.6946	0.7971	0.8478	0.8804	0.7578	0.7935	0.8284	0.854	0.8957

1	*S*_train_	0.9826	0.9649	0.961	0.9609	0.9666	0.984	0.9716	0.9723	0.9727	0.9755	0.985	0.9752	0.974	0.9735	0.9755
	*S*_test_	0.9811	0.9676	0.9643	0.9664	0.9681	0.9826	0.9716	0.9666	0.9721	0.9727	0.984	0.973	0.9723	0.9774	0.9788
	*S*_auc_	0.9335	0.9199	0.9314	0.9459	0.9539	0.9365	0.9295	0.9359	0.9552	0.9605	0.9421	0.9354	0.9492	0.9631	0.969

100	*S*_train_	0.9927	0.9851	0.9874	0.9857	0.9855	0.9949	0.9838	0.9899	0.9899	0.9894	0.9942	0.986	0.9886	0.9877	0.9899
	*S*_test_	0.9855	0.9815	0.9802	0.9766	0.9759	0.9913	0.9858	0.9811	0.9804	0.9811	0.9927	0.9865	0.9874	0.9845	0.98
	*S*_auc_	0.9535	0.9606	0.9692	0.965	0.9687	0.9749	0.971	0.9676	0.9696	0.9743	0.9869	0.9748	0.9803	0.9751	0.973

## Data Availability

The data used to support the findings of this study are available from the corresponding author upon request.

## Abbreviations

AL: Acute leukemias
ALB: Albumin
ALT: Alanine aminotransferase
AST: Aspartate aminotransferase
BASO%: Percentage of basophils
BASO#: Absolute basophil count
CL: Chronic leukemias
Cre: Creatinine
EO%: Percentage of eosinophils
EO#: Absolute eosinophil count
HCT: Hematocrit
HGB: Hemoglobin
LSVM: Linear support vector machine
LYM%: Percentage of lymphocytes
LYM#: Absolute lymphocyte count
MCH: Mean red blood cell hemoglobin
MCHC: Mean red blood cell hemoglobin concentration
MCV: Mean red blood cell volume
ML: Machine learning
MONO%: Percentage of monocytes
MPV: Mean platelet volume
NEUT%: Percentage of neutrophils
NEUT#: Absolute neutrophil count
PCT: Thrombocytocrit
PDW: Platelet distribution width
P-LCR: Platelet large cell ratio
PLT: Platelet
RBC: Red blood cell
RDW-CV: Red blood cell distribution width
RF: Random forest
SD: Standard variations
TBIL: Total bilirubin
TP: Total protein
UA: Uric acid
WBC: White blood cell.
